The article "Performance Analysis of Conventional Machine Learning Algorithms for Diabetic Sensorimotor Polyneuropathy Severity Classification Using Nerve Conduction Studies" was published in 2022. Journal: Comput Intell Neurosci.

# Performance Analysis of Conventional Machine Learning Algorithms for Diabetic Sensorimotor Polyneuropathy Severity Classification Using Nerve Conduction Studies

**DOI:** 10.1155/2022/9690940

**Published:** 2022-04-25

**Authors:** Fahmida Haque, Mamun B. I. Reaz, Muhammad E. H. Chowdhury, Serkan Kiranyaz, Sawal H. M. Ali, Mohammed Alhatou, Rumana Habib, Ahmad A. A. Bakar, Norhana Arsad, Geetika Srivastava

**Affiliations:** ^1^Department of Electrical, Electronic and System Engineering, Universiti Kebangsaan Malaysia, Bangi 43600, Selangor, Malaysia; ^2^Department of Electrical Engineering, Qatar University, Doha 2713, Qatar; ^3^Neuromuscular Division, Hamad General Hospital, Doha 3050, Qatar; ^4^Department of Neurology, Al khor Hospital, Doha 3050, Qatar; ^5^Department of Neurology, BIRDEM General Hospital, Dhaka-1000, Bangladesh; ^6^Department of Physics and Electronics, Dr. Ram Manohar Lohia Avadh University, Ayodhya 224001, India

## Abstract

**Background:**

Diabetic sensorimotor polyneuropathy (DSPN) is a major form of complication that arises in long-term diabetic patients. Even though the application of machine learning (ML) in disease diagnosis is very common and well-established in the field of research, its application in DSPN diagnosis using nerve conduction studies (NCS), is very limited in the existing literature.

**Method:**

In this study, the NCS data were collected from the Diabetes Control and Complications Trial (DCCT) and its follow-up Epidemiology of Diabetes Interventions and Complications (EDIC) clinical trials. The NCS variables are median motor velocity (m/sec), median motor amplitude (mV), median motor F-wave (msec), median sensory velocity (m/sec), median sensory amplitude (*μ*V), Peroneal Motor Velocity (m/sec), peroneal motor amplitude (mv), peroneal motor F-wave (msec), sural sensory velocity (m/sec), and sural sensory amplitude (*μ*V). Three different feature ranking techniques were used to analyze the performance of eight different conventional classifiers.

**Results:**

The ensemble classifier outperformed other classifiers for the NCS data ranked when all the NCS features were used and provided an accuracy of 93.40%, sensitivity of 91.77%, and specificity of 98.44%. The random forest model exhibited the second-best performance using all the ten features with an accuracy of 93.26%, sensitivity of 91.95%, and specificity of 98.95%. Both ensemble and random forest showed the kappa value 0.82, which indicates that the models are in good agreement with the data and the variables used and are accurate to identify DSPN using these ML models.

**Conclusion:**

This study suggests that the ensemble classifier using all the ten NCS variables can predict the DSPN severity which can enhance the management of DSPN patients.

## 1. Introduction

Diabetic sensorimotor polyneuropathy (DSPN) is one of the major complications with a prevalence of 50% that arise in patients with long-term Diabetes mellitus (DM) [1–3]. DSPN is a type of nerve damage, which can lead to many lower limb complications such as numbness, burning, pinprick sensation, and pain. In the worst case for long term DSPN, it can lead to ulceration, and amputation, suggestively increasing the chance of early death and reducing the quality of life of DM patients [4–7]. About 40 to 60 million DM patients are affected with lower limb complications because of DSPN and in every 30 seconds, one lower limb is being amputated due to DSPN [8]. Understanding the severity of this complication, early and accurate detection of DSPN is inevitable for proper treatment and to avoid severe consequences. However, diagnosis methods for the identification of DSPN patients are controversial. One study has shown that almost two-thirds of the health physicians were failed to identify the signs of DSPN, leading to misdiagnosis [9]. Even though a large number of screening and diagnosis techniques have been practiced in clinical trials and research, there is still no standardized diagnosis systems that can be globally adopted for DSPN [7, 10–12]. This is because of the variability in patterns of signs and symptoms in DSPN patients. Diagnosis of DSPN is still relied on offline interpretation by healthcare professionals. Due to the different techniques are applied in different regions of the world, this offline diagnosis is variable to the healthcare professionals, which can lead to miss leading diagnoses.

To avoid such conflict, American Diabetic Association (ADA), had issued a position statement and stated that, the diagnosis of DSPN should be based on the results from patient's clinical history and physical examination for signs and symptoms of DSPN along with nerve conduction studies (NCS) [13]. NCS has been considered as the benchmark for the identification and stratification of DSPN in clinical trials and research [1, 14]. However, it does not provide any standardized severity grading. Severity stratification of DSPN is performed using different composite scoring techniques such as neuropathy disability score (NDS), neuropathy symptom score (NSS), Toronto clinical neuropathy score (TCNS), and Michigan diabetic neuropathy score (MDNS) [15]. Even though these composite scoring techniques are easy to implement, these techniques do not provide the full diagnosis to understand the severity of the nerve damage. Henceforth, ADA recommends electrophysiological testing for accurate diagnosis of DSPN [13].

As DSPN involves the damage of the peripheral nerve, it can only be examined from the skin biopsy and sural nerve biopsy [12, 16]. However, both of these techniques are invasive and not suitable for larger clinical trials. The most studied electrophysiological examinations such as NCS, and the ophthalmic imaging tool, corneal confocal microscopy (CCM) had shown promising reliability in identifying DSPN [17–20]. CCM has shown promising performance in identifying early small fiber neuropathy and is being studied on a wide scale [21–23]. However, this technique is quite expensive as it requires expensive instruments. Moreover, it is still an under observational study for the severity classification of DSPN. NCS has long been known as the gold standard test for DSPN diagnosis [24, 25] and has been proven effective to evaluate dysfunctions of large nerve fibers [24–26]. Even though this technique has been used as a gold standard for a few decades, no severity grading system was proposed solely based on NCS. In 1994, Feldman [27], proposed a four-class severity grading system with a two-step diagnosis technique, MDNS including Michigan neuropathy screening instrument (MNSI) and NCS, however, it has not been widely used. NDS has been widely used in diabetic neuropathy-related research and is one of the most commonly used severity grading systems, however, it used only four clinical examinations of neuropathy symptoms which are not always reliable, and severe graded patients in NDS, are always referred toward NCS for better understanding [28–32]. In such a scenario, if NCS based grading system can be available, it will help the healthcare professionals to better identify and stratify DSPN patients.

The involvement of machine learning (ML) techniques in diseases diagnosis, stratification, and smart health care system are being enormously expanding due to its various advantages over traditional techniques [33–39]. Recently ML-based research for DSPN is also being focused on by the researchers. The application of ML in DSPN diagnosis using CCM has received much attention, emphasizing the automation of the CCM system for a more accurate, reliable, and reproducible diagnosis of DSPN [21, 40–42]. In literature, few works have been proposed the application of ML-based DSPN diagnosis using different composite scoring techniques like MNSI, NDS, and electrophysiological examination [2, 3, 43–45]. Barthakur et al. [46] developed artificial neural network (ANN) based DSPN diagnosis techniques using NCS with an accuracy of 99.8%. However, the result of this work could not be generalized as it has been trained on a small dataset without cross-validation. The trained ANN model is overfitted and biased, which is the reason behind the higher accuracy, and it has also only considered the median nerve for NCS. According to ADA, to diagnose patients with DSPN, at least two NCS measures should be considered abnormal. So, the NCS protocol they followed is not in compliance with ADA. Liu et al. [47] have studied the performance of ML-based facial motor NCS and found that the random forest algorithm has shown an optimal performance in differentiating normal and abnormal facial motor NCS. From this perspective, in this research, we wanted to develop different ML models, for DSPN severity classification using NCS and find out the best performing ML model for reliable severity identification of DSPN using NCS data.

In the present paper, we have investigated the performance of eight different conventional ML algorithms such as ensemble classifier (EC), random forest (RF), K-nearest neighbour (KNN), decision trees (DT), support vector machine (SVM), Naive Bayes (NB), logistic regression (LR), and discriminant analysis classifier (DAC) for severity classification of DSPN using NCS. The choice of algorithms studied in this study was based on the commonly used conventional ML algorithms in disease classification problems based on literature [3, 36, 38, 47, 48]. Ten nerve attributes have been considered for DSPN severity grading in this study. Patients were classified into four severity classes as absent, mild, moderate, and severe based on the severity grading proposed by Feldman et al. [27] using NCS. The dataset was imputed using ML techniques to deal with the missing values and different feature ranking techniques were used to rank NCS attributes. Furthermore, detailed comparisons were done to evaluate the performance of eight different algorithms and the effect of different feature ranking techniques on the performance of different ML models were also evaluated.

The novelty of this research work is the implementation and performance analysis of different conventional ML-based intelligent classifiers that will be able to classify DSPN severity levels using NCS. This study will benefit DSPN patients as well as diabetic patients with accurate, reliable, and early identification and stratification of DSPN and will help to receive early treatments to prevent severe complications like ulceration and amputation. This study investigates the effect of NCS attributes from different nerves on DSPN severity classification using feature ranking. This study can support healthcare professionals in accurate, reliable, and real-time decision making. Also, the problems due to lack of uniformity and agreements in the severity grading by different experts can be solved by using an ML-based intelligent DSPN severity classifier. As per our knowledge, this is the first study, where conventional ML learning-based models were studied for DSPN stratification using NCS variables. As NCS is considered the gold standard for DSPN diagnosis, an ML-based severity grading system will add more value to the identification and classification of DSPN. It will help the health professionals and researchers, not to depend on other secondary scoring techniques such as NDS for severity grading.

## 2. Materials and Methods

### 2.1. Data Acquisition

In this research, NCS data were collected from the Diabetes Control and Complications Trial (DCCT) and its follow up Epidemiology of Diabetes Interventions and Complications (EDIC) clinical trials which are conducted by the National Institute of Diabetes, Digestive and Kidney Diseases. DCCT enrolled 1,441 patients with type 1 diabetes in 1983 and at DCCT closeout, started EDIC with the remaining 1,375 patients from DCCT in 1994 [49–54]. The details about DCCT and EDIC patients, study protocol, inclusion and exclusion criteria, NCS criteria, NCS thresholds have been discussed by the research published by the research group [54, 55]. The NCS dataset was collected from DCCT baseline, first, second, fifth, tenth (closeout), and EDIC year thirteenth and fourteenth. Nerve conduction studies were performed by trained and certified electromyographers on the dominant side median (motor and sensory), peroneal (motor), and sural (sensory) nerves using percutaneous nerve stimulation and surface recording as done in the DCCT [54, 55]. The total dataset was consisting of 5,938 samples. The NCS variables are median motor velocity (m/sec), median motor amplitude (mV), Median Motor F-Wave (msec), Median Sensory Velocity (m/sec), Median Sensory Amplitude (*μ*V), Peroneal Motor Velocity (m/sec), Peroneal Motor Amplitude (mv), Peroneal Motor F-Wave (msec), Sural Sensory Velocity (m/sec), and Sural Sensory Amplitude (*μ*V).

### 2.2. Data Imputation

The collected NCS dataset consists of 5,938 samples, with missing values for different NCS attributes. Among the 5,938 NCS data samples, the missing number of data for each NCS attribute are as follows: median motor velocity (m/sec) 15 data, median motor amplitude (mV) 2 data, median motor F-Wave (msec) 54 data, median sensory velocity (m/sec) 128 data, median sensory amplitude (*μ*v) 12 data, peroneal motor velocity (m/sec) 48 data, peroneal motor amplitude (mv) 14 data, peroneal motor F-Wave (msec) 749 data, sural sensory velocity (m/sec) 563 data, and sural sensory amplitude (*μ*v) 33 data. The missing data were imputed with the Random forest [56] data imputation technique. Kokla et al. [56] have shown that the random forest (RF) data imputation technique outperforms other imputation techniques for medical data. Therefore, in this study, the RF technique was used for the data imputation.

### 2.3. Data Augmentation

Among the 5,938 data samples, no duplicate samples were found. The imputed NCS dataset was unbalanced. The synthetic Minority Oversampling Technique (SMOTE) technique [57] had been used to balance the training dataset to avoid data overfitting. Unlike random oversampling that only duplicates some random examples from the minority class, SMOTE generates examples based on the distance of each data (usually using Euclidean distance) and the minority class nearest neighbours, so the generated examples are different from the original minority class [58]. Python 3.7 in-house written code was used for data imputation and augmentation. In the dataset among 5,938 data samples, 2610, 1034, 1092, and 1202 samples were in absent, mild, moderate, and severe classes, respectively. 70% of the original data, 4157 (1827, 723, 764, and 841 were in the absent, mild, moderate, and severe training set) data samples were used for training while absent, mild and severe classes were augmented make the number of samples equal to absent class sample number so that all classes become equal. The remaining 30% of the original dataset, 1782 samples were used as a test set.  Figure 1 shows the number of samples in each class among the original, train, and test sets.

### 2.4. DSPN Severity Scoring for NCS

For NCS, if two or more nerve attributes are in the abnormal range, then the patients are identified as DSPN. In this study, a total of 10 NCS attributes were considered. The preprocessed NCS dataset was graded using the electrophysiological (NCS) scoring technique proposed by Feldman et al. [37]. If *x* is the number of NCS attributes, then the severity classes are divided as follows:

- Absent neuropathy: 0 ≥ *x* ≥ 1
- Mild neuropathy: *x* = 2
- Moderate neuropathy: 3 ≥ *x* ≥ 4
- Severe neuropathy: *x* ≥ 5

### 2.5. Feature Ranking

A large number of attributes may confuse the model and over-fit. Feature selections allow further dimensionality reduction. In this study, the forward feature selection approach is followed by adding 1 feature at a time and then checking the performance. To ensure using the best feature, the feature set is reordered according to feature importance. In this study, we have used three feature selection algorithms: minimum redundant maximum relevant (MRMR) [59], Feature selection using neighbourhood component analysis (fscnca) [60], and Relieff [61] algorithms.

### 2.6. Statistical Analysis

For Statistical analysis, SPSS software (version 21.0; SPSS Inc., Chicago, IL, USA) was used. All the statistical analyses for baseline characteristics of the EDIC patients were performed based on the DSPN and Non-DSPN groups and expressed as mean ± standard deviation (SD). Analysis of variance (ANOVA) was used to find out the statistical significance of the variables. An independent *t*-test was used to find out the 95% confidence intervals (95% CI). Statistical significance was considered at *p* < 0.05. Pearson's correlation coefficient was used to find out the correlation between different variables with DSPN classes. For the performance analysis of the ML models, Cohen's kappa statistic [62] was used to find the reliability of the performance of the ML models, and Matthews Correlation Coefficient (MCC) [63] was used to find the correlations between the observed and predicted classifications.

### 2.7. DSPN Severity Classifier Using NCS Variables

This study focuses on the performance analysis of different conventional ML algorithm based DSPN severity classifiers using NCS variables. Here, we trained 8 different algorithms: ensemble classifier (EC), random forest (RF), K-nearest neighbour (KNN), Decision Trees (DT), support vector machine (SVM), naive Bayes (NB), logistic regression (LR), and discriminant analysis classifier (DAC) [3, 36, 38, 47, 48]. Fitcauto function from MATLAB 2020b (The MathWorks, Inc., Natick, Massachusetts, United States) was used for training and hyperparameters' tuning of the models. We have optimized all the algorithms by using Bayesian optimization. For each algorithm, the function optimized all possible hyperparameters using Bayesian optimization [63]. After the optimization of all the algorithms, the best-performing algorithms were selected for further investigation [64]. Stratified 10-fold cross-validation was used to train and test different ML models, where the train and test dataset was divided into 70% and 30%, respectively. The training dataset was augmented to make the classes balance, while the test set was not augmented. The performance of different ML models was evaluated using a confusion matrix and different performance metrics. In this study, we use an evaluation matrix to test the ML model performance, by calculating Accuracy, Sensitivity, Specificity, F-1 Score, error rate. Receiver operating characteristic curve (ROC) and corresponding area under the curve (AUC) was generated for the best two performing models for all severity class and macro and microaverage ROC and AUC was calculated for all class.  Figure 2 illustrates the flow chart of the data processing and ML model performance analysis.

### 2.8. Validation of the Severity Grading Model with Binary DCCT/EDIC Ground Truth

In the NCS dataset, binary ground truth (Non-DSPN/Absent and DSPN) was available for the DCCT/EDIC dataset. There were 2,837 non-DSPN and 3,101 DSPN patients. Based on the severity classification, we can organize the dataset into binary classes (non-DSPN vs DSPN) and cross-validate with the DCCT/EDIC ground truth. Fisher's exact test was performed on the dataset, to find out the validity of the grading model with the ground truth by DCCT/EDIC.

## 3. Results

### 3.1. Baseline Characteristics

EDIC patients' baseline demographic variables have been observed to understand the characteristics of the patients and are shown in Table 1. The EDIC patients ages range from 20 to 50 years with an average of 35.95 ± 6.93 years, diabetic duration 14.51 ± 4.92 years. From Table 1, it can be visible that, Hemoglobin A1C (HbA1c) and low-density lipoproteins (LDL) cholesterol are not statistically significant between the DSPN and Non-DSPN classes.

### 3.2. Performance Evaluation of ML Models

NCS features were ranked based on their importance in identifying DSPN. Three different feature selection techniques were studied. In Figure 3, the results from different feature ranking techniques for NCS have been shown. The dataset was prepared based on the results from different ranking techniques and different ML models were trained using top feature combinations starting from top 1 feature, top 2 features until top 10 features. The optimized hyperparameters for ML models used in this study are listed in Table 2. Tables 3–5 summarize the best performance by different ML models for three different feature ranking techniques.

From Tables 3–5, it can be observed that the ensemble model with all NCS features (10) using the relief feature ranking technique is exhibiting better performance with an accuracy of 93.40%, sensitivity of 91.77%, and specificity of 98.44% in comparison to other models.  Figure 4 shows the confusion matrix of the entire test set for the ensemble model classifier using all 10 features by relief feature ranking technique.

The random forest (RF) model exhibits the second-best performance using all 10 features with an accuracy of 93.26%, sensitivity of 91.95%, and specificity of 98.95%. From the MCC, it can be observed that EC, RF, and DT show a strong correlation (range 0.87–0.90) between the predicted and the true class for all feature ranking techniques. However, for the rest of the models, the MCC values are in the range of 0.58–0.69 indicating that the predicted and the true classes are weakly correlated. Figures 5 and 6 depict the ROC for the best performing two algorithms. From Figure 5, it can be observed that the microaverage and macroaverage AUCs are 0.96 and 0.95, respectively, and the AUC for each class for the best performing model has been shown.

The impact of individual features on DSPN severity has also been studied. The best-performing model was trained for individual NCS features. EC model was trained for all 10 NCS variables and the performance metrics for all the features can be found in Table 6. It can be observed that individual features are unable to contribute to identifying DSPN severity with better performance. This also indicates that all the NCS features are contributing to DSPN severity identification in combination. So, with the available features, it becomes possible to the best possible stratification performance using the best ML model.

### 3.3. Validation of the Severity Grading Model with Binary DCCT/EDIC Ground Truth

Considering the reasonable performance of the proposed 4-class classification problem, it is important to evaluate the model performance with any existing ground truth as the class labels of the 4-class NCS dataset is not widely adopted classification scheme and are not used in any machine learning paradigm. Therefore, our proposed model could be more reliable than Feldman's classification. However, this has to be validated. In the NCS dataset, a binary ground truth (non-DSPN vs DSPN) was available for the DCCT/EDIC dataset, which is reliable ground truth labels. We, therefore, tested the performance of our model for two-class (DSPN (mild, moderate and severe) vs non-DSPN (absent) classification. Fisher's exact test was performed on the dataset, to find out the validity of the grading model with the ground truth by DCCT/EDIC.  Table 7 shows the number of samples in different classes graded by the model proposed by Feldman et al. [27] in comparison to DCCT/EDIC ground truth. It was found that all the absent patients were accurately identified by the grading model proposed by Feldman et al. [27].

However, among the 2837 non-DSPN, 219 and 8 patients were classified in Mild and Severe classes, respectively (Table 7). On the contrary, using our proposed stratification model, only 42 non-DSPN patients were miss-classified to DSPN and 52 Mild DSPN patients were miss-classified to non-DSPN. Overall, 3.8% miss-classification of Feldman et al. [27] model is reduced to 1.6% using our model.

## 4. Discussion

Diabetic sensorimotor polyneuropathy (DSPN) is a length-dependent impediment for diabetes patients. Over the past decades, research is being conducted to establish DSPN definitions, diagnosis criteria, standardized diagnosis method, and treatment protocol [1, 4, 13, 65]. However, to date, DSPN diagnosis and severity stratification rely on subjective analysis of the diagnosis results by specialized expertise. As there are controversies among health professionals regarding the DSPN screening criteria and variation in screening techniques in different countries, subjective diagnosis can be misleading.

American Diabetic Association (ADA) had issued a position statement in 2017 and stated that diagnosis of DSPN should be based on the results from patient's clinical history and physical examination for signs and symptoms of DSPN along with nerve conduction studies (NCS) [13]. NCS has been considered as the benchmark for the identification and stratification of DSPN [1, 14]. However, it does not provide any severity grading. In practice, severity stratification of DSPN is performed using different composite scoring techniques. Even though these composite scoring techniques are widely studied, their reliability to understand the severity of the nerve damages is questionable. Henceforth, ADA recommends NCS testing for accurate diagnosis of DSPN [13] and it has long been known as the gold standard test for DSPN diagnosis [66]. Nerve conduction study has been proven effective to evaluate dysfunctions of large nerve fibers [66]. Even though this technique has been used as a gold standard for a few decades, a standardized severity grading system for NCS is not available. In 1988, Dyck et al. [66] proposed a 4 stages, severity grading system for DSPN, where they considered NCS, neurological examination, and quantitative nerve test. In 1994, Feldman et al. [27], proposed a four-class severity grading system with a two-step diagnosis technique [67], MDNS including Michigan neuropathy screening instrument (MNSI) and NCS. In 1997, Dyck et al. [68] proposed a composite scoring technique including 4 stage severity grading which combines the Neuropathy Impairment Score–Lower Limb (NIS-LL) with seven tests (NIS(LL)+7). Among the seven tests, vibration detection threshold, peroneal nerve compound muscle action potential amplitude, motor conduction velocity and distal motor latency, tibial distal motor latency, and sural sensory nerve action potential amplitude were included. In 2015, a Japanese group led by Baba et al. [69] proposed a new NCS based 5 class severity grading system using the attributes from the tibial motor and sural sensory nerves. However, this grading model has been validated on the Japanese population, and for type 2 diabetes patients. England et al. [65] suggested observing sural sensory and peroneal motor nerve attributes as these nerves are the most sensitive for DSPN diagnosis. Besides, if any of the attributes from these two nerves are abnormal, other nerve attributes are recommended to be studied, which includes the tibial nerve. In the grading system by Baba et al. [69], however, the peroneal nerve was not considered, hence its performance in diagnosing DSPN is debatable.

In 2020, Weng et al. [70] used a 4-class severity grading based on 5 nerve conduction studies for DSPN stratification, where if patients have 2 abnormal NCS among 5, it is graded as mild, 3-4 abnormal NCS is graded as moderate and greater than equal to 5 abnormal NCS is considered as severe. This is proposed as electrophysiological severity definition by Feldman et al. [27]. This grading system has been used in our study for comparing the performance of the ML models with NCS data for DSPN severity classification. In the NCS dataset, binary ground truth (non-DSPN/absent and DSPN) was available for DCCT/EDIC. Fisher's exact test was performed on the dataset, to find out the validity of the grading model with the ground truth by DCCT/EDIC.

We found that there is a grey area between the absent class and mild class by the ground truth and the grading model proposed by Feldman et al. [27]. 21% of the original Absent class patients were identified as Mild class. As these two are adjacent classes, having a grey area is quite common in clinical work as these adjacent classes share almost similar or slightly different NCS values. ML can be a potential solution to distinguish these minor characteristic changes in adjacent classes and accurately identify the classes. However, in this research, we used the grading model proposed by Feldman et al. [27] for comparison, as apart from the grey zone for mild class, it is in agreement with the DCCT/EDIC ground truth for the other three classes.

Recently, ML-based research for DSPN is being focused on by the researchers. In literature, few works have been proposed the application of ML-based DSPN diagnosis using different composite scoring techniques like MNSI, NDS, and electrophysiological examination [2, 3, 43–45]. In the present paper, we have investigated the performance of eight different conventional ML algorithms such as ensemble classifier (EC), random forest (RF), K-nearest neighbour (KNN), Decision Trees (DT), support vector machine (SVM), naive Bayes (NB), logistic regression (LR), and discriminant analysis classifier (DAC) for severity classification of DSPN using NCS. Ten nerve attributes have been considered for DSPN severity grading in this study. Patients were classified into four severity classes as absent, mild, moderate, and severe based on the severity grading proposed by Feldman et al. [27].

Three different feature ranking techniques such as relief, mrmr, and fscnca were used to find out the best performing NCS features in DSPN severity grading, while all the ML models were optimized using the Bayesian optimization technique. The optimized ML models were trained for different combinations of features starting from Top 1 to Top 10 features depending on different feature ranking results. For all three feature ranking techniques, the ensemble classification model has shown better performance in comparison with other ML models used in this study. The best performance was achieved by the EC model with all 10 NCS features using the relief feature ranking technique with an accuracy of 96.33%. It was evident from Tables 3–5 that for all the feature ranking techniques, the EC model has superior performance while all the NCS parameters are used.

From Cohen's Kappa statistic for different ML models, we have found that KNN, SVM, NB, LR, and DAC exhibited fair agreement between the predicted and expected classes with a kappa value range from 0.21–0.45, indicating that, the inputs are fairly accurate to identify DSPN severity using these models. For the EC, RF, and DT, the kappa value ranged from 0.77–0.82, which indicates that the models are in good agreement [62] with the data and the variables used and are perfectly accurate to identify DSPN using these ML models [62]. Now to understand the impact of individual NCS features, we have trained the best performing ensemble model from the previous analysis for each NCS variable. It was observed that none of the NCS variables was capable of identifying DSPN severity classes with better performance individually. From this study, we can recommend that all NCS variables (available in this dataset) need to be considered while DSPN severity grading for higher accuracy of the model's performance. From this observation, it can be said that all the NCS features combined were contributing better to identifying DSPN. Therefore, any other NCS datasets with more NCS parameters can be optimized with better-ranked features to enhance the model performance even further. As per our knowledge, this is the first study, where conventional ML learning-based models were studied for DSPN severity classification using NCS variables. The strength of our study was it has been designed based on a large cohort of patients from 28 different medical centers of EDIC trials, which adds value to our developed model by having variability in the population. However, we have considered the database consists of only type 1 diabetic patients. In the future, both type 1 and 2 patients' datasets can be incorporated to have a realistic and generalized model in DSPN severity classification using NCS. The ML models need to be validated on multiple datasets for classification problems [71]. In this study, the ML models were developed and tested on the dataset collected from DCCT and EDIC clinical trials. In a clinical disease classification problem, having multiple datasets, where clinical data from patients are used are not always available publicly, especially for the large clinical trials like used in this study. However, as the ML models, were trained on larger real clinical trials data, and the ground truths have been provided by validated clinical professionals, the development and testing of the ML models performance can be considered reliable. In future, the ML model's performance needed to be validated with a different dataset. As the NCS model has been selected as a gold standard, an ML-based severity grading system will add more value to the identification and classification of DSPN. It will help the health professionals and researchers, not to depend on other secondary scoring techniques such as NDS for severity grading.

## 5. Conclusions

DSPN is being considered to have a life-threatening impact on diabetes patients since the 1980s. Even though much research is being conducted, still now, DSPN diagnosis techniques are complicated contradictory, and subjective. Nerve conduction studies (NCS) have been used as a gold standard for DSPN for over a few decades. Many researchers have proposed many grading systems over the year, however, none has been adopted as a standardized severity grading model for NCS. An ML-based grading system can help to approximate the versatility of the available grading methods and improve the performance in accurately and reliably identifying DSPN severity.

We have observed the performance of different conventional ML algorithms in the diagnosis and severity stratification of DSPN using NCS. We have used different feature ranking techniques to find out the best combination of features for DSPN identification and stratification. From this analysis, we have found that the optimized ensemble classifier algorithm with all NCS variables provides the best performance in DSPN stratification. Here we noticed that feature ranking techniques have no impact on the feature selection from the NCS dataset, indicating that, all the variables are equally important and combining them will help in identifying different DSPN classes. So, an ensemble classifier based NCS grading technique can help healthcare professionals to identify DSPN patients and grade their severity. This type of system can overcome the problem of inconsistency and lack of agreement between professionals with diagnostic criteria for DSPN.

## Figures and Tables

**Figure 1:** Number of samples in classes among the original, train, and test datasets.

**Figure 2:** Flow chart of the data processing and ML model performance analysis for DSPN severity classification using NCS data.

**Figure 3:** Ranking of the NCS features using (a) mrmr (b) relief (c) fscnca feature ranking techniques.

**Figure 4:** Confusion matrix of the test set for ensemble classifier using Top 10 ranked features by relief feature ranking technique.

**Figure 5:** ROC curve for all 10 features using relief feature ranking using ensemble classifier.

**Figure 6:** ROC curve for all 10 features using fscnca feature ranking using random forest classifier.

**Table 1:** Baseline characteristics of the EDIC patients.

*N* = 1255	Mean	Std. error mean	Min	Max	95% confidence interval		*r*	*p*	*f*
					Lower limit	Upper limit			
Age (years)	35.95 ± 6.93	0.20	20.42	50.99	35.57	36.34	0.18	<0.05	43.96
Diabetic duration (years)	14.51 ± 4.92	0.14	7.08	26.92	14.24	14.78	0.12	<0.05	18.40
Hba1c (%)	8.22 ± 1.39	0.04	0.00	14.00	8.14	8.30	0.10	0.95	12.54
HDL Cholesterol (mg/dl)	52.559 ± 15.98	0.45	0.00	103.0	51.67	53.44	0.002	<0.05	0.01
LDL Cholesterol (mg/dl)	110.68 ± 36.48	1.03	0.00	235.0	108.7	112.7	0.07	0.21	5.62
BMI (kg/m^2^)	26.17 ± 4.05	0.11	16.63	39.48	25.94	26.39	0.04	<0.05	1.56
Hypertension (%)	0.23 ± 0.42	0.01	1.00	0.16	0.20	0.25	0.16	<0.05	31.75

**Table 2:** Optimized Hyperparameters of the studied ML algorithms.

Algorithm	Tuned Hyperparameters
Discriminant analysis classifier (DAC)	Discriminate type = quadratic
	FillCoeffs = Off

Ensemble classification model (EC)	Method = AdaBoostM2
	Number of learning cycles = 477
	Learning rate = 0.9845217666852848
	Maximum number splits = 311,
	Number of variables to sample = all

K-nearest neighbour (KNN) model	Distance = Euclidean,
	Number of neighbors = 1,
	Distance weight = inverse
	Standardized = false

Naive Bayes classifier (NB)	Distribution names = mvmn (multivariate multinomial distribution)
	Kernel = normal
	Support = unbounded

Support vector machine classifier (SVM)	Learners = SVM
	Categorical predictors = all
	Split criterion = deviance
	Maximum number splits = 960
	Surrogate = off

Decision Tree (DT)	Split criterion = deviance
	Maximum number splits = 960
	Surrogate = off

Random Forest (RF)	Number of trees = 100
	Compute OOB prediction (flag to compute out-of-bag predictions) = on
	Method = classification

Logistic Regression (LR)	lambda (regularization parameter) = 1e-4

**Table 3:** Performance evaluation of different ML models using mrmr feature selection technique for NCS.

	Features	Accuracy (%)	Sensitivity (%)	Specificity (%)	F1-score (%)	Error rate	MCC	Kappa	AUC
EC	Top 10	93.25 ± 0.95	91.69 ± 1.03	98.44 ± 0.61	91.77 ± 1.02	0.07 ± 0.01	0.90	0.82	1.00
RF	Top 10	93.06 ± 0.63	91.61 ± 0.69	98.92 ± 0.59	91.52 ± 0.76	0.07 ± 0.01	0.89	0.81	1.00
DT	Top 10	91.34 ± 1.60	89.86 ± 1.88	99.37 ± 0.46	89.46 ± 1.99	0.09 ± 0.02	0.87	0.77	0.98
KNN	Top 10	79.47 ± 0.94	75.71 ± 0.89	91.95 ± 1.05	75.89 ± 1.01	0.21 ± 0.01	0.69	0.45	0.91
SVM	Top 8	75.98 ± 1.59	69.29 ± 1.92	75.18 ± 2.06	72.54 ± 1.84	0.24 ± 0.02	0.64	0.36	0.96
NB	Top 10	73.90 ± 2.02	72.35 ± 2.16	95.31 ± 1.01	72.43 ± 2.02	0.26 ± 0.02	0.64	0.30	0.95
LR	Top 9	71.76 ± 1.89	69.45 ± 1.85	93.42 ± 1.22	69.19 ± 1.82	0.28 ± 0.02	0.60	0.25	0.95
DAC	Top 9	70.73 ± 2.44	68.66 ± 2.43	94.11 ± 1.24	68.52 ± 2.24	0.29 ± 0.02	0.59	0.22	0.94

**Table 4:** Performance evaluation of different ML models using relief feature selection technique for NCS.

	Features	Accuracy (%)	Sensitivity (%)	Specificity (%)	F1-score (%)	Error rate	MCC	Kappa	AUC
EC	Top 10	93.40 ± 0.97	91.77 ± 1.15	98.44 ± 0.73	91.90 ± 1.11	0.07 ± 0.01	0.90	0.82	1.00
RF	Top 10	93.25 ± 0.80	91.92 ± 1.04	99.10 ± 0.53	91.78 ± 1.04	0.07 ± 0.01	0.90	0.82	1.00
DT	Top 10	91.43 ± 1.66	89.99 ± 1.96	99.40 ± 0.47	89.57 ± 2.05	0.09 ± 0.02	0.87	0.77	0.98
KNN	Top 10	79.47 ± 0.94	75.71 ± 0.89	91.95 ± 1.05	75.89 ± 1.01	0.21 ± 0.01	0.69	0.45	0.91
SVM	Top 8	75.98 ± 1.59	69.29 ± 1.92	75.18 ± 2.06	72.54 ± 1.84	0.24 ± 0.02	0.64	0.36	0.96
NB	Top 10	73.90 ± 2.02	72.35 ± 2.16	95.31 ± 1.01	72.43 ± 2.02	0.26 ± 0.02	0.64	0.30	0.95
LR	Top 9	71.76 ± 1.89	69.45 ± 1.85	93.42 ± 1.22	69.19 ± 1.82	0.28 ± 0.02	0.60	0.25	0.95
DAC	Top 9	70.73 ± 2.44	68.66 ± 2.43	94.11 ± 1.24	68.52 ± 2.24	0.29 ± 0.02	0.59	0.22	0.94

**Table 5:** Performance evaluation of different ML models using fscnca feature selection technique for NCS.

	Features	Accuracy (%)	Sensitivity (%)	Specificity (%)	F1-score (%)	Error rate	MCC	Kappa	AUC
RF	Top 10	93.26 ± 0.91	91.95 ± 1.03	98.95 ± 0.62	91.80 ± 1.07	0.07 ± 0.01	0.90	0.82	1.00
EC	Top 10	93.16 ± 0.89	91.49 ± 1.00	98.38 ± 0.78	91.62 ± 0.96	0.07 ± 0.01	0.89	0.82	1.00
DT	Top 10	91.60 ± 1.95	90.19 ± 2.36	99.40 ± 0.47	89.78 ± 2.44	0.08 ± 0.02	0.87	0.78	0.98
KNN	Top 10	79.47 ± 0.94	75.71 ± 0.89	91.95 ± 1.05	75.89 ± 1.01	0.21 ± 0.01	0.69	0.45	0.91
SVM	Top 8	75.03 ± 1.42	68.17 ± 1.76	72.69 ± 2.70	71.95 ± 1.65	0.25 ± 0.01	0.63	0.33	0.95
NB	Top 10	73.90 ± 2.02	72.35 ± 2.16	95.31 ± 1.01	72.43 ± 2.02	0.26 ± 0.02	0.64	0.30	0.95
LR	Top 10	71.57 ± 1.92	69.15 ± 1.88	93.33 ± 1.27	68.91 ± 1.84	0.28 ± 0.02	0.59	0.24	0.95
DAC	Top 10	70.33 ± 2.09	68.15 ± 2.04	93.96 ± 1.42	68.05 ± 1.95	0.30 ± 0.02	0.58	0.21	0.93

**Table 6:** Performance evaluation of individual NCS features using the EC model.

NCS Features	Accuracy (%)	Sensitivity (%)	Specificity (%)	F1-score (%)	Error rate	MCC	kappa
Peroneal motor velocity (m/sec)	57.09 ± 1.30	57.00 ± 1.29	55.49 ± 1.16	56.24 ± 1.22	0.43 ± 0.01	0.42	0.13
Median sensory velocity (m/sec)	48.54 ± 1.22	48.44 ± 1.21	46.46 ± 1.39	47.43 ± 1.29	0.51 ± 0.01	0.30	0.27
Median motor F-wave (msec)	55.92 ± 1.62	55.84 ± 1.62	55.14 ± 1.65	55.48 ± 1.63	0.44 ± 0.02	0.41	0.15
Peroneal motor amplitude (mV)	50.27 ± 1.57	50.17 ± 1.56	47.74 ± 1.65	48.92 ± 1.60	0.50 ± 0.02	0.33	0.25
Sural sensory velocity (m/sec)	51.11 ± 1.25	51.00 ± 1.25	48.26 ± 1.55	49.59 ± 1.40	0.49 ± 0.01	0.34	0.23
Median motor velocity (m/sec)	53.53 ± 1.39	53.44 ± 1.38	51.40 ± 1.44	52.40 ± 1.41	0.46 ± 0.01	0.37	0.19
Median sensory amplitude (*μ*V)	49.84 ± 1.65	49.72 ± 1.64	46.29 ± 2.00	47.94 ± 1.83	0.50 ± 0.02	0.32	0.25
Peroneal motor F-wave (msec)	52.92 ± 0.90	52.84 ± 0.91	51.37 ± 1.09	52.09 ± 0.98	0.47 ± 0.01	0.37	0.20
Sural sensory amplitude (*μ*V)	50.15 ± 1.07	50.03 ± 1.06	47.30 ± 1.25	48.63 ± 1.15	0.50 ± 0.01	0.32	0.25
Median motor amplitude (mV)	42.73 ± 1.92	42.65 ± 1.93	39.93 ± 2.11	41.25 ± 2.03	0.57 ± 0.02	0.22	0.34

**Table 7:** Validation of the grading model proposed by Feldman et al. [27] and this work with DCCT/EDIC ground truth using Fisher exact test.

	DCCT/EDIC ground truth		Total no of samples in the dataset
	Non-DSPN	DSPN	
*Severity grading by Feldman et al.* [27]			
Absent	2610 (100%)	0 (0%)	2610
Mild	219 (21%)	815 (79%)	1034
Moderate	0 (0%)	1092 (100%)	1092
Severe	8 (0.67%)	1194 (99.33%)	1202
Total	2837	3101	5939

*Severity grading by this work*			
Absent	2568 (98.4%)	42 (1.61%)	2610
Mild	52 (5.03%)	982 (94.97%)	1034
Moderate	0 (0%)	1092 (100%)	1092
Severe	0 (0%)	1202 (100%)	1202
Total	2837	3101	5939

## Data Availability

The database is available on request from the National Institute of Diabetes and Digestive and Kidney Diseases (NIDDK) websites. Diabetes Control and Complications Trial/Epidemiology of Diabetes Interventions and Complications (DCCT/EDIC) database: https://repository.niddk.nih.gov/studies/edic/.
